# Cerebrolysin™ efficacy in a transgenic model of tauopathy: role in regulation of mitochondrial structure

This article has been retracted.

**DOI:** 10.1186/1471-2202-15-90

**Published:** 2014-07-21

**Authors:** Edward Rockenstein, Kiren Ubhi, Margarita Trejo, Michael Mante, Christina Patrick, Anthony Adame, Philipp Novak, Marion Jech, Edith Doppler, Herbert Moessler, Eliezer Masliah

**Affiliations:** Department of Neurosciences, University of California San Diego, La Jolla, CA USA; Clinical Research & Pharmacology, EVER Neuro Pharma GmbH, Unterach, Austria; Department of Pathology, University of California San Diego, La Jolla, CA USA

**Keywords:** Tau, GSK3β, Drp-1, Neuroprotection, Alzheimer’s disease, Tauopathies

## Abstract

**Background:**

Alzheimer’s Disease (AD) and Fronto temporal lobar dementia (FTLD) are common causes of dementia in the aging population for which limited therapeutical options are available. These disorders are associated with Tau accumulation. We have previously shown that Cerebrolysin^TM^ (CBL), a neuropeptide mixture with neurotrophic effects, ameliorates the behavioral deficits and neuropathological alterations in amyloid precursor protein (APP) transgenic (tg) mouse model of AD by reducing hyper-phosphorylated Tau. CBL has been tested in clinical trials for AD, however it’s potential beneficial effects in FTLD are unknown. For this purpose we sought to investigate the effects of CBL in a tg model of tauopathy. Accordingly, double tg mice expressing mutant Tau under the mThy-1 promoter and GSK3β (to enhance Tau phosphorylation) were treated with CBL and evaluated neuropathologically.

**Results:**

Compared to single Tau tg mice the Tau/GSK3β double tg model displayed elevated levels of Tau phosphorylation and neurodegeneration in the hippocampus. CBL treatment reduced the levels of Tau phosphorylation in the dentate gyrus and the degeneration of pyramidal neurons in the temporal cortex and hippocampus of the Tau/GSK3β double tg mice. Interestingly, the Tau/GSK3β double tg mice also displayed elevated levels of Dynamin-related protein-1 (Drp-1), a protein that hydrolyzes GTP and is required for mitochondrial division. Ultrastructural analysis of the mitochondria in the Tau/GSK3β double tg mice demonstrated increased numbers and fragmentation of mitochondria in comparison to non-tg mice. CBL treatment normalized levels of Drp-1 and restored mitochondrial structure.

**Conclusions:**

These results suggest that the ability of CBL to ameliorate neurodegenerative pathology in the tauopathy model may involve reducing accumulation of hyper-phosphorylated Tau and reducing alterations in mitochondrial biogenesis associated with Tau.

## Background

The cognitive deficits in patients with Alzheimer’s Disease (AD) and Fronto-temporal lobar degeneration (FTLD) are associated with selective loss of neuronal populations in the neocortex, limbic system and subcortical nuclei, in association with progressive accumulation of the cytoskeletal protein Tau [1–7]. FTLD is an heterogenous group of neurodegenerative disorders that are characterised by atrophy of the frontal and/or temporal lobes [8]. Examples of FTLD include Pick’s disease (PiD) and corticobasal degeneration. In contrast to AD, which presents predominantly with memory loss, FTLD is associated with changes in personal and social conduct, behaviour and language disturbances, and often motor symptoms [9]. In FTLD neurodegeneration is associated with either aggregated Tau or aggregated TAR DNA-binding protein of 43 kDa (TDP-43), fused-in-sarcoma or yet unidentified proteins in affected brain regions in the absence of overt beta-amyloid (Aβ) plaques [10].

The mechanisms through which aggregated and hyperphosphorylated Tau leads to neurodegeneration in AD and FTLD are not completely clear. Recent studies suggest that abnormal Tau might mediate neurodegeneration by dysregulating Dynamin-related protein-1 (Drp-1), which in turns results in alterations in mitochondria biogenesis [11]. Moreover, Tau phosphorylation at Ser262 through PAR-1 contributes to Tau-mediated neurodegeneration under a pathological condition in which axonal mitochondria are depleted [12, 13]. Thus Tau dependent loss of axonal mitochondria may play an important role in the toxicity and pathogenesis of AD [12]. Tau also mediates the neurotoxic effects of Aβ which can promote the mis-localization of tau to the dendrites [14] and mitochondria [15]. In contrast, Tau reduction has been shown to ameliorate the behavioral and neurodegenerative pathology in models of AD [16]. Therefore strategies directed at reducing Tau accumulation might be protective for AD and FTLD.

We have previously shown that in APP transgenic (tg) mice over expressing the amyloid precursor protein (APP), CBL reduces synaptic and behavioral deficits [17–19]. CBL is a peptide mixture with neurotrophic-like effects that improves cognition in patients with mild to moderate AD [20–22]. Moreover, a recent double-blind trial of CBL was demonstrated to improve the activities of daily living and psychiatric deficits in patients with moderate to moderately severe AD [21]. Several other randomized double-blind studies in patients with AD have shown that CBL is consistently superior to placebo at reducing cognitive alterations [23–25].

CBL also ameliorates the neurodegenerative pathology and accumulation of Tau in a combined APP tg mouse model injected with AAV2-Tau [26]. We have recently shown that CBL might reduce APP and Tau pathology in models of AD by decreasing CDK5 and GSK3β activity [26]. However, it is unclear whether CBL might ameliorate the neurodegenerative pathology in models of FTLD. For this purpose we generated a new cross of the mutant Tau tg mice expressing human 4 repeat Tau (4R-Tau), bearing the missense mutations V337M and R406W, under the mThy-1 promoter [27] with GSK3β tg mice. The Tau/GSK3β double tg model displays biochemical and neuropathological features reminiscent of tauopathies including elevated levels of Tau phosphorylation and neurodegeneration. We found that administration of CBL reduces the levels of Tau and ameliorates the neurodegeneration in this Tau/GSK3β double tg model and this is accompained by reduced levels of Drp-1 and mitochondrial pathology associated with Tau.

## Results

### Neuropathological and biochemical alterations in Tau/GSK3β tg mice

The parental single Tau mutant tg mice that we use have been reported to display moderate alterations in tau accumulation [27], additionally, previous studies have shown that adding GSK3β enhances the pathology [28], therefore Tau/GSK3β bigenic mice were generated by crossing Tau tg mice expressing human Tau under the mThy-1 promoter with GSK3β tg mice in order to enhance tau phosphorylation. These double tg mice were subsequently used to evaluate the effects of CBL. Immunochemical analysis was performed in order to compare the expression patterns and distribution of tau and GSK3β between the single Tau tg and the Tau/GSK3β tg mice. By western blot levels of total GSK3β (t-GSK3β) were 3 fold higher in the GSK3β and Tau/GSK3β tg compared to non-tg and Tau tg mice (Figure 1A, B). Likewise, levels of phosphorylated GSK3β (p-GSK3β) were 3-fold higher in the GSK3β and Tau/GSK3β tg compared to non-tg and Tau tg mice (Figure 1A, B). GSK3β was phosphorylated at the T-loop tyrosine Y216 which could play a role in forcing open the substrate-binding site and has been proposed to correlate with kinase activation. Levels of Total-Tau (t-Tau) were 2–3 fold higher in the Tau tg and the Tau/GSK3β tg mice compared to non-tg and GSK3β tg (Figure 1A, C). Levels of phosphorylated Tau (p-Tau, AT8, Ser202/Thr205) were increased by 40% in the GSK3β tg, by 200% in the Tau tg and by 350% in the Tau/GSK3β tg compared to non-tg (Figure 1A, C). The levels of p-Tau were significantly different between the Tau tg and the Tau/GSK3β tg. Immunocytochemical analysis showed that in the GSK3β tg and Tau/GSK3β tg mice levels of GSK3β immunoreactivity were higher in the pyramidal cell in neocortex, CA1-CA3 and dentate gyrus of the hippocampus (Figure 1D, E), as well as in neurons in the basal ganglia and brain-stem (data not shown), compared to the non-tg controls and Tau tg mice. These same neuronal populations also displayed increased p-Tau immunoreactivity in the neocortex and granular cells in the hippocampus with the AT8 antibody (Figure 1F, G). The levels of p-Tau were significantly higher in the Tau/GSK3β tg compared to the Tau tg mice (Figure 1F, G).

To further investigate the effects of age on Tau pathology in the single and bigenic mice, immunocytochemical analysis with p-Tau (AT8) antibody was performed in mice at 3, 6 and 12 months of age. The non-tg and GSK3β tg mice display low levels of p-Tau immunoreactivity at the 3 time points (Figure 2A, B). Compared to the control, the Tau tg mice displayed a mild increase in p-Tau at 6 m and 12 m of age (Figure 2A, B). The Tau/GSK3β tg displayed a mild increase in p-Tau at 3 m and a robust progressive increase in p-Tau at 6 m and 12 m of age (Figure 2A, B). Tau/GSK3β tg mice displayed greater p-Tau compared to single Tau tg mice therefore for subsequent studies with CBL we compared the effects on non-tg vs bigenic mice.

**Figure 1:** **Characterization of Tau/GSK3β bigenic mice. (A)** Representative immunoblot image for total GSK3β (t-GSK3β), phospho-GSK3β (p-GSK3β)(Y216), total Tau (t-Tau) and phospho-Tau (p-Tau) levels in the hippocampus of the Tau/GSK3β bigenic mice compared to Tau tg, GSK3β tg and non-tg mice. Actin was used as a loading control. **(B)** Analysis of levels of t-GSK3β and p-GSK3β showing 3 fold higher levels in GSK3β bigenic mice. **(C)** Analysis of levels of t-Tau and p-Tau (AT8) showing higher levels of p-Tau in bigenic mice compared to Tau tg mice. **(D,** **E)** Immunohistochemical and image analysis of pGSK3β immunoreactivity in the dentate gyrus of the hippocampus (inset) in the non-tg, single tg and Tau/GSK3β bigenic mice. **(F,** **G)** Immunohistochemical and image analysis of p-Tau (AT8) immunoreactivity in the dentate gyrus of the hippocampus (inset) in the non-tg, single tg and Tau/GSK3β bigenic mice The boxes indicate regions shown at higher magnification in the lower panels. Scale bar in upper panel = 250 μm, in lower panels = 30 μm. Error bars represent mean ± SEM (n = 6 per group, 6 m/o). *Indicates a significant difference (p < 0.05) between non-tg and single or bigenic mice analyzed by one-way ANOVA and Dunnett’s post hoc test. # Indicates a significant difference (p < 0.05) between Tau tg and bigenic mice analyzed by one-way ANOVA and Tukey-Krammer post hoc test.

**Figure 2:** **Comparison of effects of aging on p-Tau in non-tg single tg and Tau/GSK3β bigenic mice. (A)** Representative images of immunohistochemical analysis with the p-Tau (AT8) in the neocortex and hippocampus in the non-tg, single tg and Tau/GSK3β bigenic mice at 3, 6 and 12 months of age. **(B)** Image analysis of optical density in the hippocampus represented as a line graph in the non-tg, single tg and Tau/GSK3β bigenic mice at 3, 6 and 12 months of age. Scale bar = 250 μm, in lower panels = 250 μm. Error bars represent mean ± SEM (n = 6 per age and genotype).

### Chronic treatment with CBL reduces Tau phosphorylation in the bigenic mice

Non-tg and bigenic mice were treated for 3 months (beginning at 3 months of age) with CBL and brains were analyzed with p-tau antibodies. Mice were 6 month old at the time of the analysis. By immunoblot, levels of t-Tau were elevated in the Tau/GSK3β bigenic mice compared to the non-tg, no effects of CBL administration on t-Tau were observed (Figure 3A-D). Likewise levels of p-Tau species as detected with the AT8 and AT270 antibodies were increased in the Tau/GSK3β tg compared to non-tg, however in Tau/GSK3β tg mice treated with CBL, the levels of p-Tau were reduced by 50% compared to the vehicle-treated Tau/GSK3β tg group (Figure 3A, E).

Immunohistochemical analysis showed that p-Tau immunoreactivity was more prominent in the hippocampal CA1 and dentate gyrus (DG) regions of the Tau/GSK3β bigenic mice compared to non-tg controls (Figure 3E, F). Tau/GSK3β tg mice treated with CBL displayed a 40% decrease in the levels of p-Tau immunostaining in the hippocampus compared to the Tau/GSK3β tg vehicle group (Figure 3E, F).

**Figure 3:** **Immunoblot and immunocytochemical analysis of effect of CBL on Tau in Tau/GSK3β bigenic mice. (A)** Representative Immunoblot image of total-tau (t-Tau), phospho-Tau (p-Tau) at epitopes recognized by the AT8 (Ser202/Thr205) and AT270 (Thr181) antibodies and actin levels in vehicle and CBL treated Tau/GSK3β bigenic mice in comparison to non-tg mice. **(B-** **D)** Image analysis of levels of t-Tau, p-Tau (AT8) and p-Tau (AT270) respectively in vehicle and CBL treated Tau/GSK3β bigenic mice in comparison to non-tg mice. **(E)** Immunohistochemical analysis of p-Tau (AT8) immunoreactivity in the hippocampus of vehicle and CBL treated Tau/GSK3β bigenic mice in comparison to non-tg mice. Boxes in upper panels are represented at higher magnification in the lower panels. **(F)** Image analysis of p-GSK3β immunoreactivity in the hippocampus of vehicle and CBL treated Tau/GSK3β bigenic mice in comparison to non-tg mice. **(A, C)** Scale bar in upper panels = 250 μm, in lower panels = 50 μm. **(B, D)** Error bars represent mean ± SEM (n = 6 per group, 6 m/o). *Indicates a significant difference (p < 0.05) between vehicle and CBL treated Tau/GSK3β bigenic mice analyzed by one-way ANOVA and Dunnett’s post hoc test.

### Neuroprotective effects of CBL in the Tau/GSK3β bigenic mice

Next we evaluated whether the effects of CBL in the bigenic mice ameliorated the neurotoxic effects of p-Tau. For this purpose vibratome sections were immunolabeled with antibodies against the dendritic marker- MAP2 and the pan-neuronal marker- NeuN. Vehicle-treated Tau/GSK3β bigenic mice displayed a significant 25-30% reduction in MAP2 immunoreactivity in the CA1 region and the DG molecular layer compared to the vehicle treated non-tg controls (Figure 4A-C). In contrast, bigenic mice treated with CBL showed levels of MAP2 immunoreactivity comparable to non-tg controls (Figure 4A-C). Stereological analysis of neuronal cell density with NeuN showed that the vehicle treated Tau/GSK3β bigenic mice displayed a significant 35-40% reduction in NeuN immunoreactivity cells in the CA1 region and the DG granular cell layer compared to the vehicle treated non-tg controls (Figure 4D-F). Treatment with CBL ameliorated loss of NeuN positive cells in the Tau/GSK3β bigenic mice, which showed cell counts comparable to those observed in the non-tg controls (Figure 4D-F).

**Figure 4:** **Effect of CBL on neuropathological alterations in Tau/GSK3β bigenic mice. (A)** Immunohistochemical analysis of dendritic pathology as evidenced by MAP2 immunoreactivity in the hippocampus of vehicle and CBL treated Tau/GSK3β bigenic mice in comparison to non-tg mice. Boxes in upper panels are represented at higher magnification in the lower panels. **(B)** Quantitative analysis of MAP2 immunoreactivity in the CA1 region of the hippocampus of vehicle and CBL treated Tau/GSK3β bigenic mice in comparison to non-tg mice. **(C)** Quantitative analysis of MAP2 immunoreactivity in the molecular layer (ML) of the dentate gyrus of the hippocampus of vehicle and CBL treated Tau/GSK3β bigenic mice in comparison to non-tg mice. **(D)** Immunohistochemical analysis neuronal density as evidenced by NeuN immunoreactivity in the hippocampus of vehicle and CBL treated Tau/GSK3β bigenic mice in comparison to non-tg mice. Boxes in upper panels are represented at higher magnification in the lower panels. **(E)** Quantitative analysis of NeuN immunoreactivity in the CA1 region of the hippocampus the hippocampus of vehicle and CBL treated Tau/GSK3β bigenic mice in comparison to non-tg mice. **(F)** Quantitative analysis of NeuN immunoreactivity in the molecular layer of the dentate gyrus of the hippocampus of vehicle and CBL treated Tau/GSK3β bigenic mice in comparison to non-tg mice. **(A,** **D)** Scale bar in upper panels = 250 μm, in lower panels = 50 μm. **(B,** **C,** **E,** **F)** Error bars represent mean ± SEM (n = 6 per group, 6 m/o). *Indicates a significant difference (p < 0.05) between vehicle and CBL treated Tau/GSK3β bigenic mice analyzed by one-way ANOVA and Dunnett’s post hoc test.

### *Treatment with CBL reverses alterations in Drp-1 in Tau/*GSK3β *bigenic mice*

Previous studies have shown that Tau neurotoxicity might be mediated by alterations in mitochondrial biogenesis [11], in this context we examined the levels of Drp-1 a protein involved in mitochondrial fission and the general mitochondrial marker Tom40 [29] in the bigenic mice. By immunoblot analysis, Drp-1 was identified as a single band at approximately 80 kDa (Figure 5A). Compared to the vehicle treated non-tg controls, the vehicle treated Tau/GSK3β bigenic mice displayed a significant 35-40% increase in Drp-1 in the cytosolic fraction from hippocampal homogenates (Figure 5A, B). In contrast, bigenic mice treated with CBL showed levels of Drp-1 lower than those detected in the vehicle treated bigenic mice. Moreover, levels of Drp-1 in the CBL-treated bigenic mice were slightly below the levels of the non-tg controls (Figure 5A, B). Level of phosphorylated Drp-1 (p-Drp-1) were higher in the vehicle-treated Tau/GSK3β bigenic mice in comparison to vehicle- and CBL-treated non-tg mice (Figure 5C). CBL treatment significantly decreased expression of p-dDrp-1 in the Tau/GSK3β bigenic mice, bringing it to levels more comparable with non-tg controls (Figure 5C).

Immunocytochemical analysis showed that Drp-1 reactivity was abundant in the neuropil of the cortex. Likewise, Tom40 immunoreactivity was most abundant in the neuropil displaying a fine punctate pattern (Figure 5D). Compared to the vehicle treated non-tg controls, the vehicle treated Tau/GSK3β bigenic mice displayed a significant 30-35% increase in Drp-1 and Tom40 immunoreactivity, while the bigenic mice treated with CBL showed levels of Drp-1 and Tom40 similar those observed in the non-tg controls (Figure 5D-F).

**Figure 5:** **Effect of CBL on mitochondrial proteins in Tau/GSK3β bigenic mice. (A)** Immunoblot analysis of Drp-1 levels in hippocampal homogenates from vehicle and CBL treated Tau/GSK3β bigenic mice in comparison to non-tg mice. Actin was used as a loading control. **(B)** Quantitative analysis of Drp-1 levels in the hippocampus of vehicle and CBL treated Tau/GSK3β bigenic mice in comparison to non-tg mice. **(C)** Quantitative analysis of p-Drp-1 levels in the hippocampus of vehicle and CBL treated Tau/GSK3β bigenic mice in comparison to non-tg mice. **(D)** Immunohistochemical analysis of Drp-1 and Tom40 levels in the hippocampus of vehicle and CBL treated Tau/GSK3β bigenic mice in comparison to non-tg mice. Arrows indicate immunoreactive mitochondria. **(E)** Quantitative analysis of Drp-1 levels in the hippocampus of vehicle and CBL treated Tau/GSK3β bigenic mice in comparison to non-tg mice. **(F)** Quantitative analysis of Tom40 levels in the hippocampus of vehicle and CBL treated Tau/GSK3β bigenic mice in comparison to non-tg mice. Scale Bars = 5 μm, Error bars represent mean ± SEM (n = 6 per group, 6 m/o). *Indicates a significant difference (p < 0.05) between vehicle non-tg mice and vehicle-treated Tau/GSK3β bigenic mice and # indicates a significant difference (p < 0.05) between vehicle and CBL treated Tau/GSK3β bigenic mice analyzed by one-way ANOVA and Dunnett’s post hoc test.

### *CBL ameliorates the mitochondrial alterations in Tau/*GSK3β *bigenic mice*

Given that the neurodegenerative pathology in the Tau/GSK3β bigenic mice was concomitant with an increase in Drp-1, and p-Drp-1, expression and Tom40 puncta, we next sought to determine whether these alterations correspond to mitochondrial alterations. For this purpose electron microscopic analysis was performed in hippocampal sections. Remarkably, compared to the vehicle and CBL-treated non-tg mice (Figure 6A), the vehicle-treated Tau/GSK3β bigenic mice showed extensive mitochondrial alterations including presence of lamellar intra-mitochondrial inclusions, incompletely divided and fragmented mitochondria (Figure 6B, D-F). In contrast, the mitochondria from the CBL treated bigenic mice were similar to controls (Figure 6C-F). Consistent with these observations, image analysis showed that in the vehicle treated Tau/GSK3β bigenic mice the proportion of small (less than 0.5 μm), dividing mitochondria with inclusions was greater when compared to the non-tg controls, while bigenic mice treated with CBL displayed mitochondrial characteristics similar to non-tg controls (Figure 6D-E).

**Figure 6:** **Ultrastructural analysis of mitochondrial structure in Tau/GSK3β bigenic mice. (A)** Ultrastructural analysis of mitochondrial structure in vehicle-treated and CBL treated non-tg mice. **(B)** Ultrastructural analysis of mitochondrial structure in vehicle-treated Tau/GSK3β bigenic mice, boxes in upper panel are shown at a higher magnification in the lower panels. **(C)** Ultrastructural analysis of mitochondrial structure in CBL-treated Tau/GSK3β bigenic mice. **(D)** Quantitative analysis of number of small mitochondria (less than 5 μm) in vehicle and CBL treated Tau/GSK3β bigenic mice in comparison to non-tg mice. **(E)** Quantitative analysis of number of dividing mitochondria in vehicle and CBL treated Tau/GSK3β bigenic mice in comparison to non-tg mice. **(F)** Quantitative analysis of number of mitochondrial inclusions in vehicle and CBL treated Tau/GSK3β bigenic mice in comparison to non-tg mice. Scale Bar = 0.5 μm, error bars represent mean ± SEM (n = 6 per group, 6 m/o). *Indicates a significant difference (p < 0.05) between vehicle non-tg mice and vehicle-treated Tau/GSK3β bigenic mice and # indicates a significant difference (p < 0.05) between vehicle and CBL treated Tau/GSK3β bigenic mice analyzed by one-way ANOVA and Dunnett’s post hoc test.

## Discussion

The present study showed that the Tau/GSK3β double tg model displays biochemical and neuropathological features reminiscent of tauopathies such as elevated levels of Tau phosphorylation and hippocampal neurodegeneration. Interestingly, the Tau/GSK3β double-tg mice also display elevated levels of Drp-1, p-Drp-1, and increased fragmentation of mitochondria accompanied by abnormal divisions and membranous inclusions. In the bigenic mice, CBL treatment reduced the accumulation of p-Tau, ameliorated the neurodegenerative pathology, decreased Drp-1 and p-Drp-1 expression, and returned mitochondria to characteristics comparable to non-tg mice.

The mThy1-Tau (V337M and R406W) tg model has been shown to accumulate soluble p-Tau in the limbic system and to display spatial learning impairments [27]. The FTDP-17 R406W tau mutation has been described in an American, a Dutch, and a Japanese family [30–32]. To enhance these deficits we crossed these animals with an mThy1-GSK3β tg model. This resulted in more widespread accumulation of p-Tau and neurodegeneration in the hippocampus. The alterations in the Tau/GSK3β double tg model are comparable to previous reports using a tg model with conditional overexpression of GSK3β in forebrain neurons [33, 34].

Given the findings with the age dependent analysis showing that p-Tau accumulation is more abundant in Tau/GSK3β double tg compared to the single tg mice, we decided to test the effects of CBL in the bigenic mice. Animals were treated beginning at 3 months of age for 3 months, because at the earlier age group the Tau pathology was subtler, becoming progressively worse at 6 and 12 months of age. Therefore, the effects described in our study represent a preventive trial study for CBL. Future study will be needed testing the effects of Cerebrolysin in older Tau/GSK3β double tg compared to single Tau tg mice. Moreover, future studies in other models of Tauopathy such as the Tg4510 are warranted to further validate our observations.

An additional novel finding of our model was the presence of widespread mitochondrial pathology and increased Drp-1 expression. This is consistent with recent studies showing that accumulation of Tau might lead to neurodegeneration via alterations in mitochondrial biogenesis [11, 35–37]. Drp-1 is known to promote mitochondrial fission, consistent with this our ultra-structural studies showed increased in fragmented mitochondria with abnormal divisions and inclusions. Remarkably, hyperactivation of kinases that phosphorylate Tau such as CDK5 and GSK3β has been shown to interfere with Drp-1 function leading to mitochondrial alterations [38, 39], and GSK3β has been reported to phosphorylate Drp-1 [40]. In these bigenic mice, treatment with CBL ameliorated the neurodegenerative pathology, decreased p-Tau, reduced Drp-1 and normalized mitochondrial morphology. The mechanisms through which CBL might achieve these effects on the bigenic model are not completely clear. We have previously shown that this neurotrophic peptide mixture is capable of reducing the behavioral deficits in APP tg mouse model of AD-like pathology [17, 18] by blocking CDK5 and GSK3β [41], resulting in decreased APP maturation and Aβ biosynthesis [41], increased neurogenesis [42] and synaptic formation [18, 41]. Therefore, it is possible that the effects on Drp-1 observed in the bigenic mice might be partially mediated by the inhibitory effects of CBL on CDK5 and GSK3β [43]. Moreover, and consistent, with the present study, treatment with CBL in APP tg injected with AAV2-Tau has been reported to result in a significant amelioration of neurodegenerative pathology and decreased levels of Tau phosphorylation at critical sites dependent on GSK3β and CDK5 activity [26]. These results suggest that CBL administration may have some therapeutic efficacy for the treatment of tauopathies.

## Conclusions

In the Tau/GSK3β double tg model CBL may rescue the deficits by reducing tau hyperphosphorylation, which in turn may restore mitochondrial biogenesis. These results suggest that CBL’s ability to rescue neurodegenerative pathology in the tauopathy model may involve reducing accumulation of hyper-phosphorylated Tau and then restoring altered mitochondrial biogenesis associated with Tau. Therefore, CBL might be of potential therapeutical value in the treatment of certain forms of FTLD.

## Methods

### *Generation of double mutant Tau and*GSK3β*Tg Mice and CBL treatment*

For these experiments, tg mice expressing the human 4R Tau mutated (V337M and R406W) under the control of the mThy-1 promoter (mThy1-Tau) (line 441) [27]. These mice display memory deficits and a moderate increase in tau phosphorylation in the neocortex and limbic system. To enhance the Tau pathology the mThy1-tau tg were crossed with mice over-expressing human GSK3β under the control of the mThy-1 promoter (mThy1- GSK3β). This line of mice expresses high levels of constitutive active GSK3β that can hyper-phosphorylate Tau and other substrates. We have previously generated similar GSK3β tg mouse lines with both dominant negative and constitutively active effects [44]. Genomic DNA was extracted from tail biopsies and analyzed by PCR amplification, as described previously [45]. Transgenic lines were maintained by crossing heterozygous tg mice with non-transgenic (non tg) C57BL/6 × DBA/2 F1 breeders. All mice were heterozygous with respect to the transgene. A total of 24 Tau/GSK3β tg mice (3 month (m) old; n = 12 CBL treated and n = 12 saline) and 24 non tg mice (3 m old; n = 12 CBL treated and n = 12 saline) were utilized. A subset of single tg mThy1-Tau tg and mThy1- GSK3β were utilized as controls. Mice were injected daily with saline alone or CBL (i.p., 5 ml/kg) for a total of 3 months. The last injection of vehicle or CBL was administered 24 hrs before sacrificing the animals. CBL is a mixture of peptides and amino acids obtained after high quality hydrolyzing and purification from porcine brain, more information is available at the web site (http://www.hypermed.com.au/Clinical%20Research/EVER2010_Monograph_screen.pdf). CBL was a gift from EverPharma. An additional group of un-treated non-tg, single tg and bigenic mice were utilized for analysis of effects of aging at 3, 6 and 12 months of age (n = 6 per genotype/age group). All experiments described were approved by the animal subjects committee at the University of California at San Diego (UCSD) and were performed according to NIH guidelines for animal use.

### Tissue processing

In accordance with NIH guidelines for the humane treatment of animals, mice were anesthetized with chloral hydrate and flush-perfused transcardially with 0.9% saline. Brains were removed and divided sagitally. The left hemibrain was post-fixed in phosphate-buffered 4% paraformaldehyde (pH 7.4) at 4°C for 48 hr and sectioned at 40 μm with a Vibratome 2000 (Leica, Germany), while the right hemibrain was snap frozen and stored at −70°C for protein analysis.

### Immunohistochemical analysis

For this purpose as previously described [26, 29], blind-coded 40 μm thick vibratome sections were immunolabeled with the mouse monoclonal antibodies against Drp-1 (1:500, Santa Cruz), Tom40 (1:1000, Santa Cruz), synaptophysin (presynaptic terminal marker, 1:40, Chemicon), GFAP (astroglial marker, 1:1000, Chemicon), p-Tau (AT8, 1:500, Pierce; AT270 1:500, Pierce), t-Tau (1:500, Dako), t-GSK3β (1:500, Cell Signaling) and p-GSK3β (GSK3βY216, 1:500, Life Technologies), as previously described [18, 41]. After overnight incubation with the primary antibodies, sections were incubated with Texas red or FITC-conjugated horse anti-mouse IgG secondary antibody (1:75, Vector Laboratories), transferred to SuperFrost slides (Fisher Scientific) and mounted under glass coverslips with anti-fading media (Vector). All sections were processed under the same standardized conditions. The immunolabeled blind-coded sections were imaged with the laser-scanning confocal microscope (LSCM, MRC1024, BioRad) and analyzed with the Image 1.43 program (NIH), as previously described [18]. To confirm the specificity of primary antibodies, control experiments were performed where sections were incubated overnight in the absence of primary antibody (deleted) or preimmune serum and primary antibody alone.

The numbers of NeuN-immunoreactive neurons were estimated using unbiased stereological methods [46]. Hemi-sections containing the neocortex, hippocampus and striatum were outlined using an Olympus BX51 microscope running StereoInvestigator 8.21.1 software (Micro-BrightField). Grid sizes for the striatum, frontal cortex, and hippocampal CA3 pyramidal layer were: 900 × 900, 800 × 800, and 300 × 300 μm, respectively, and the counting frames were 40 × 40, 30 × 30, and 50 × 50 μm, respectively. The average coefficient of error for each region was 0.9. Sections were analysed using a 100 × 1.4 PlanApo oil-immersion objective. A 5-μm high disector, allowed for 2 μm top and bottom guard-zones.

### Immunoblot analysis

Briefly, as previously described [47] protein homogenates from the hippocampus of vehicle and CBL-treated Tau/GSK3β bigenic mice and non-tg mice were prepared by fractionation into cytosolic and membrane-bound constituents. Twenty micrograms of cytosolic protein per mouse were loaded onto 4-12% Bis-Tris (Invitrogen) SDS-PAGE gels, transferred onto Immobilon membranes, washed and blocked in BSA. After an overnight incubation with antibodies against total (1:1000, Cell Signaling) or p-GSK3β (Y216, 1:1000, Life Technologies) [33, 34], total (1:500, Dako) and p-Tau AT8, AT270 (1:1000, Pierce) and Drp-1 (1:500, Santa Cruz), membranes were incubated in appropriate secondary antibodies, reacted with ECL and developed on a VersaDoc gel-imaging machine (Bio-Rad, Hercules, CA). Anti-beta-actin (1:1000; Sigma) antibody was used to confirm equal loading.

### Electron microscopy and immunogold analysis

Briefly [48], vibratome sections were post-fixed in 1% glutaraldehyde, treated with osmium tetraoxide, embedded in epon araldite and sectioned with the ultramicrotome (Leica, Germany). Grids were analyzed for mitochondrial morphology [49] with a Zeiss OM 10 electron microscope as previously described [40]. Electron micrographs were obtained at a magnification of 25,000X.

### Statistical analysis

Analyses were carried out with the StatView 5.0 program (SAS Institute Inc., Cary, NC). Differences among means were assessed by one-way ANOVA with post-hoc Dunnett’s. Comparisons between 2 groups were assessed using the two-tailed unpaired Student's t-test. Correlation studies were carried out by simple regression analysis and the null hypothesis was rejected at the 0.05 level.

## Abbreviations

4R-Tau: Four-repeat tau
AAV2: Adeno-associated virus sub-type-2
AD: Alzheimer’s disease
APP: Amyloid precursor protein
ANOVA: Analysis of variance
Aβ: Amyloid beta protein
CDK5: Cyclin-dependent kinase 5
CBL: CBL
DG: Dentate gyrus
DNA: Deoxyribonucleic acid
Drp-1: Dynamin-related protein-1
FITC: Fluorescein isothiocyanate
FTLD: Fronto-temporal lobar degeneration
GCL: Granular cell layer of the dentate gyrus
GFAP: Glial fibrillary acidic protein
GSK3β: Glycogen synthase kinase 3-beta
GTP: Guanosine-5’-triphosphate
MAP2: microtubule-associated protein-2
ML: Molecular layer of the dentate gyrus
N: Number
NIH: National institutes of health
p-GSK3b: Phosphorylated glycogen synthase kinase 3-beta
p-Tau: Phosphorylated tau
PCR: Polymerase chain reaction
PiD: Pick’s disease
SDS-PAGE: Sodium dodecyl sulfate- polyacrylamide gel electrophoresis
t-GSK3β: Total glycogen synthase kinase 3-beta
t-Tau: Total tau
TDP43: TAR DNA-binding protein of 43 kDa
Tg: Transgenic
UCSD: University of California, San Diego.
